# Targeting GSTP1-dependent ferroptosis in lung cancer radiotherapy: Existing evidence and future directions

**DOI:** 10.3389/fmolb.2022.1102158

**Published:** 2022-12-16

**Authors:** Xin Tan, Xiang Huang, Baolong Niu, Xingdong Guo, Xiao Lei, Baolin Qu

**Affiliations:** ^1^ Department of Radiation Oncology, The First Medical Center of Chinese PLA General Hospital, Beijing, China; ^2^ Medical School of Chinese PLA, Beijing, China

**Keywords:** ferroptosis, radiotherapy, lung cancer, GSTP1, mechanism

## Abstract

Radiotherapy is applied in about 70% patients with tumors, yet radioresistance of tumor cells remains a challenge that limits the efficacy of radiotherapy. Ferroptosis, an iron-dependent lipid peroxidation regulated cell death, is involved in the development of a variety of tumors. Interestingly, there is evidence that ferroptosis inducers in tumor treatment can significantly improve radiotherapy sensitivity. In addition, related studies show that Glutathione S-transferase P1 (GSTP1) is closely related to the development of ferroptosis. The potential mechanism of targeting GSTP1 to inhibit tumor cells from evading ferroptosis leading to radioresistance has been proposed in this review, which implies that GSTP1 may play a key role in radiosensitization of lung cancer *via* ferroptosis pathway.

## 1 Background

Lung cancer is a malignancy with the highest mortality rate, with no treatment method that could effectively prolong the long-term survival rate of lung cancer patients (Sung et al., 2021). Therefore, finding ways to improve the survival rate of lung cancer patients has become the current focus in clinical research. Radiotherapy is a common treatment method for lung cancer and plays an increasingly important role. With the development of precision radiotherapy technology, the efficacy of radiotherapy and its status in tumor treatment have significantly increased (Santivasi and Xia, 2014). Although radiotherapy is the main method of tumor treatment, it produces unsatisfactory therapeutic results. These poor outcomes are diverse in pattern and associated with DNA repair, cell energetics, gene mutations, complex tumor microenvironment and immune response meditated by radiotherapy. All of the above factors ultimately contribute to tumor resistance to radiotherapy (Raghav et al., 2012; Buckley et al., 2020; Chandra et al., 2021; Busato et al., 2022). Currently, radioresistance has become one of the leading causes of treatment failure in lung cancer patients. Ferroptosis is an iron-dependent form of cell death marked by excessive accumulation of lipid peroxides, which is significantly different from apoptosis, necroptosis and autophagy in morphology, genetic and biochemical characteristics fields (Dixon et al., 2012). The discovery of ferroptosis has led to new insights into tumor therapy, in which it has been found that ferroptosis might be involved in radiotherapy-induced cell death (Lang et al., 2019; Lei et al., 2020a; Ye et al., 2020). Glutathione S-transferase P1 (GSTP1) is a member of the glutathione-S-transferase (GST) family, which is capable of detoxifying cells from endogenous and exogenous toxic compounds by using glutathione (GSH) or by acting as a ligand (Mian et al., 2016). Studies have shown that GSTP1 plays a crucial role in maintaining cellular oxidative homeostasis and regulating cell proliferation and apoptosis (Holley et al., 2007). In addition, it has been surprisingly found that GSTP1 is involved in tumor development through ferroptosis pathway (Tew et al., 2011). Therefore, exploring the interaction of GSTP1 and ferroptosis in tumor radioresistance may provide us with a new approach to tumor radiosensitization. In this review, we discuss recent research advances on the role of ferroptosis and GSTP1 in lung cancer radiotherapy.

## 2 The potential role and its mechanisms of ferroptosis in radiotherapy

The mechanism of ferroptosis involves a confrontation between the intracellular ferroptosis execution system and the ferroptosis defense system. When the cellular activity promoting ferroptosis significantly exceeds the antioxidant buffering capacity provided by the ferroptosis defense system, there is an excessive accumulation of lipid peroxides on the cell membrane and subsequent membrane rupture, leading to cellular ferroptosis (Stockwell et al., 2020; Zheng and Conrad, 2020). The damage to the cellular structure by radiotherapy is mainly divided into two ways: direct way and indirect way. The direct way is mainly the direct action of high energy X-rays on the DNA double strand of the cell, causing it to break and inducing cell cycle arrest, senescence and cell death (Baskar et al., 2012). In addition to direct damage to DNA, ionizing radiation can also act on organisms through indirect effects. For example, after absorption of ionizing radiation by living cells, ionizing radiation can cause cellular damage by generating chemicals such as reactive oxygen species (ROS) (Azzam et al., 2012; Santivasi and Xia, 2014; Pouget et al., 2018). However, multiple tumors have evolved strategies to avoid cell death, such as loss of TP53 tumor suppressor function, increased expression of antiapoptotic regulators (Bcl-2, Bcl-xL) or survival signals (Igf1/2), thus exhibiting radioresistance to radiotherapy, which undoubtedly one of the main factors affecting patient outcome as well as prognosis (Hanahan and Weinberg, 2011). The concept of ferroptosis, first proposed by Prof. Stockwell’s team in 2012, is a regulated cell death process caused by excessive accumulation of iron ions and reactive oxygen species-induced dysregulated accumulation of cellular lipid peroxidation metabolism (Dixon et al., 2012; Stockwell et al., 2017). It is morphologically characterized by mitochondrial wrinkling and a decrease in the number of mitochondrial cristae, an increase in membrane density and thickness, insignificant morphological changes in the nucleus (Stockwell et al., 2017). It is characterized by excessive accumulation of lipid peroxides and is closely associated with intracellular iron overload, free radical production, fatty acid supply and lipid peroxidation (Li et al., 2020; Stockwell, 2022). Radiotherapy can induce ferroptosis in the specified cancers through several pathways as following.

### 2.1 Radiotherapy might affect ferroptosis through iron metabolism

Iron overload is associated with the development of lung cancer, and there is a significant positive correlation between high iron intake and lung cancer risk. Datas from a clinical trial show that serum iron, ferritin and total iron binding are significantly higher in lung cancer patients than in healthy controls (Sukiennicki et al., 2019). The higher the serum iron concentration, the greater the risk of developing lung cancer (Sukiennicki et al., 2019; Ward et al., 2019). Under normal conditions, extracellular iron bounding to transferrin to form a complex is mediated by transferrin receptor 1 (TfR1) on the cell membrane into the intracellular compartment, where it is converted to ferrous ions by ferric reductase and subsequently stored in the intracellular unstable iron pool *via* the divalent metal transporter protein divalent metal transporter 1 (DMT1), and the excess iron ions are stored as inert iron in ferritin in the cell, maintaining intracellular iron homeostasis (Masaldan et al., 2018; Lei et al., 2020a). When iron ions are overloaded, the iron ions entering the cell react with reactive oxygen species in the Fenton reaction, peroxidizing polyunsaturated fatty acids on the cell membrane and generating lipid peroxides, leading to damage of the cell membrane structure and eventually triggering cell death (Conrad and Proneth, 2019). Under ionizing radiation and oxidative stress or certain other pathological conditions, iron homeostasis can be severely altered. This alteration can manifest itself in several ways, one of which is an increase in intracellular levels of potentially harmful unstable iron pools leading to oxidative membrane damage and cell death of cells (Aroun et al., 2012). Therefore, radiotherapy may also affect the occurrence of ferroptosis by modulating iron metabolism. Ivanov et al. significantly improved the efficiency of radiotherapy in glioma-bearing mice by adding mineralized iron water to the tumor-bearing animals, which reduced monocytes and tumor volume in glioma-bearing mice under radiotherapy. Further addition of iron chelators weakened the tumor suppressive effect of radiotherapy because of blocking radiation-induced ferroptosis (Ivanov et al., 2013; Ivanov et al., 2015). Qin et al. found all-lactoferrin Holo-Lf was able to increase the expression of transferrin receptor, ferritin and ferroregulin, indicating increased iron uptake, storage and output, combined with radiotherapy could promote ROS production and increase lipid peroxidation end product malondialdehyde (MDA), thereby enhancing ferroptosis in MDA-MB-231 cells (Zhang et al., 2021a). Sato et al. shown that mitochondrial dysfunction increased intracellular H_2_O_2_, Fe^2+^ levels and might lead to increased production of -OH, resulting in lipid peroxidation and ferroptosis (Takashi et al., 2020). Zheng et al. found that the deubiquitinating enzyme USP35 regulated ferroptosis in lung cancer by targeting FPN (Tang et al., 2021a). Jun et al. disclosured that in ischemia-reperfusion-treated rat hearts, ubiquitin-specific protease seven could increase iron uptake and thus promoted ferroptosis by activating p53 leading to upregulation of TfR1 (Tang et al., 2021b). Tomita K et al. unfolded that miR⁃7⁃5p could impede Fe^2+^ transport into mitochondria by inhibiting mitoglobin under radiation, leading to the onset of intracellular hydroxyl radical levels and Fenton reaction-induced cytoplasmic membrane oxidation, ultimately causing radiation-induced ferroptosis (Tomita et al., 2019). In addition, Jaewang Lee et al. found that PCBP1, as a ferric ion chaperone protein, could inhibit iron-mediated ferritin phagocytosis and lipid peroxidation and was an important regulator of ferroptosis. Further experiments demonstrated that downregulation of PCBP1 increased the sensitivity of head and neck cancer to ferroptosis (Lee et al., 2022). In addition, many other researchers found that radiotherapy might affect ferroptosis by mediating the expression of iron metabolism-related proteins such as iron ion-related carriers like ferritin, FPN, regulatory iron regulators, membrane iron transport auxiliary protein (Hephaestin) and copper cyanobacteria by mediating hypoxia-inducible factor 1α (HIF-1α) or HIF-2α (Shah et al., 2009; Singhal et al., 2021; Yang et al., 2022). Therefore, we consider that the regulation of intracellular iron ion content by radiation to cause iron overload to enhance ferroptosis sensitivity in tumor cells is expected to be an effective way to enhance radiosensitivity.

### 2.2 Radiotherapy induces ferroptosis by promoting lipid peroxidation

Hyperoxidation of phospholipids containing polyunsaturated fatty acids (PUFA-PL) catalyzed by iron is the core feature of ferroptosis. Lipid peroxidation of PUFA generates a variety of oxidation products. Among them, lipid hydroperoxides (LOOHs) are the initial products of peroxidation. The secondary products are aldehydes, of which MDA and 4-hydroxynonenal (4-HNE) are the most abundant (Feng and Stockwell, 2018). Yang et al. finds that ferroptosis can be driven by peroxidation of polyunsaturated fatty acids (PUFA) at the diallyl site, which is pretreated with PUFA containing the heavy hydrogen isotope deuterium (D-) at the peroxidation site. Pretreatment of cells with PUFA containing the heavy hydrogen isotope deuterium (D-PUFA) at the peroxidation site prevents PUFA peroxidation and ferroptosis (Yang et al., 2016). Therefore, the content of intracellular PUFAs determines the degree of lipid peroxidation and the susceptibility of cells to ferroptosis (Lei et al., 2021a). Driven by the highly reactive OH • radicals generated by the Fenton reaction and the presence of a large amount of the bis-allylic, PUFA are the most susceptible to damage by exposure to high doses of radiation. In contrast, monounsaturated fatty acids (MUFA) are less susceptible to peroxidation due to the absence of the bis-allylic, which could inhibit lipid peroxidation and ferroptosis by replacing polyunsaturated fatty acids in the cell membrane (Feng and Stockwell, 2018). Therefore, cancer cells can be sensitized to ferroptosis by modulating the activities of enzymes involved in MUFA-PL synthesis, such as SCD1 and ACSL3. Polyunsaturated fatty acids containing diallyl provide substrates that are peroxidized to drive ferroptosis (Tesfay et al., 2019; Zou et al., 2020). Acyl coenzyme A synthase long chain family member 4 (ACSL4) esterifies CoA to free fatty acids, especially polyunsaturated fatty acids, and radiotherapy can collectively promote lipid peroxidation and ultimately ferroptosis by generating large amounts of ROS and upregulating the expression of the key enzyme ACSL4. In addition, knockdown of the ACSL4 gene in tumor cells leads to significant radioresistance (Doll et al., 2017; Lei et al., 2020a). Meanwhile, radiation is able to significantly increase the staining of C11-BODIPY, lipid peroxidation markers MDA and 4-HNE in cancer cells and tumor samples, indicating that radiation induces lipid peroxidation (Lei et al., 2020a; Zhang et al., 2021a; Zhou et al., 2022). Similarly, irradiated cells exhibit increased expression of the ferroptosis marker gene prostaglandin endoperoxide synthase 2 (PTGS2) (Busato et al., 2022; Yang et al., 2022). Furthermore, Seiji Torii et al. shows that knockdown of Arachidonate 15-Lipoxygenase (ALOX15) decreases erastin-induced and RSL3-induced cellular ferroptosis, on the contrary exogenous overexpression of ALOX15 enhances the effects of these compounds. This suggests that LOX-catalyzed lipid hydroperoxide production in the cell membrane promotes tumor ferroptosis (Shintoku et al., 2017). In contrast, treatment with baicalin (ALOX15 inhibitor) after irradiation restores normal levels of systemic irradiation-induced inflammatory cytokines and improves survival in mice (Thermozier et al., 2020). Dixon and Angeli et al. finds that the free radical scavenger statin Ferrostatin and the lipid peroxidase inhibitor/fat-soluble antioxidant vitamin E, among other lipophilic antioxidants and iron chelator drugs can modulate the occurrence of cellular ferroptosis by inhibiting the process of lipid peroxidation (Dixon et al., 2012; Angeli et al., 2017). Therefore, it is reasonable to assume that radiotherapy can influence the onset of ferroptosis by mediating the biosynthesis of polyunsaturated fatty acids in cell membranes to promote the accumulation of lipid peroxides.

### 2.3 Radiotherapy induces ferroptosis by depleting GSH and inhibiting the synthesis of GPX4

Glutathione which is synthesized from glycine, glutamate and cysteine is an important non-enzymatic antioxidant for intracellular scavenging of ROS, and its metabolic balance is closely related to the regulation of ferroptosis. Glutathione peroxidase 4 (GPX4) as a selenoperoxidase is a key upstream regulator of ferroptosis which plays two simultaneous roles, one in converting reduced GSH to glutathione disulfide (GSSG) and the other is to inhibit ferroptosis by reducing phospholipid hydroperoxides (PLOOHs) to the corresponding alcohols (PLOHs), thereby preventing the accumulation of lipid peroxides (Jiang et al., 2021). The cysteine-glutamate reverse transporter (System-Xc) is a dimer composed of the transporter-active transmembrane protein solute carrier family seven member 11(SLC7A11) and the transmembrane regulatory protein solute carrier family three member 2 (SLC3A2), in which cysteine is the rate-limiting precursor for GSH synthesis. Inhibition of SystemXc-function can lead to GSH depletion and indirectly affect the ability of GPX4 to catalyze lipid peroxide reduction reactions, resulting in ROS accumulation and triggering ferroptosis (Yang et al., 2016). Zou et al. finds that Interferon (IFNγ) secreted by CD8^+^ T cells and ATM activated by radiotherapy can synergistically inhibit SLC7A11 expression to limit cystine uptake by tumor cells, leading to reduced GSH synthesis and thus promoting lipid peroxidation and ferroptosis (Lang et al., 2019). Wang et al. finds that RBMS1 inhibits SLC7A11 translation, reduces SLC7A11-mediated cystine uptake and promotes ferroptosis in lung cancer cells (Zhang et al., 2021b). Cobler et al. finds that inhibition of SLC7A11 after Erastin treatment increases radiosensitivity in SLC7A11^+^ breast cancer cells *in vitro* and *in vivo*, while it has no effect on SLC7A11^-^ cancer cells, this process accompanied by a decrease in intracellular GSH synthesis that promotes cell death (Cobler et al., 2018). Li finds that nuclear factor erythroid 2-related factor 2 (NRF2) can inhibit radiation-induced ferroptosis by regulating SLC7A11 in esophageal squamous cell carcinoma (ESCC), promoting radioresistance in ESCC (Feng et al., 2021). Ye LF finds that ferroptosis is a mechanism of radiation-induced cancer cell death. When tumors have evolved specific resistance mechanisms such as a resistant state susceptible to GPX4 inhibition and ferroptotic cell death, the combination of ferroptosis inducers and radiotherapy has potential applications in cancers, especially those who have undergone EMT (Ye et al., 2020). In addition, Yu et al. finds that knockdown of GPX4 can reduce radiotherapy resistance in NSCLC cells by inducing ferroptosis (Pan et al., 2019). Gao et al. confirms that knockdown Ribonucleotide reductase subunit M1 (RRM1) promotes the occurrence of radiation-induced lipid peroxidation, decreases GSH levels, increases GSSH levels and elevates MDA levels. It is believed that targeting RRM1 can disrupt the antioxidant resistance system of tumor cells to mediate the onset of ferroptosis and thus radiosensitize tumor cells (Gao et al., 2022). Thus we have the same expectations for GSTP1. Shibata et al. also demonstrates the radiosensitizing effect of erastin on lung adenocarcinoma cells NCI-H1975 and tumor xenograft models accompanied by lower levels of glutathione (Shibata et al., 2019). Therefore, inhibition of the GSH/GPX4 pathway by SLC7A11 in combination with radiotherapy induces ferroptosis in tumor cells has strong application. When such ferroptosis inducers act as a radiosensitizer, in addition to the DNA double-strand damage effect, more ROS can be generated in tumor cells through other additional pathways, thus aggravating lipid peroxidation and cell death. In addition, there may be other regulatory mechanisms for the maintenance of intracellular GSH/GPX4 homeostasis, further studies targeting other influences on this pathway to induce ferroptosis and enhance radiosensitivity provide a broad scope for exploration.

## 3 GSTP1 as a potential regulator in radiotherapy of cancer

Radiotherapy exerts its anti-tumor effects mainly by generating oxidative stress (Mukha et al., 2021), thus oxidative stress-related enzymes may affect the effect of radiotherapy in cancer patients. Enzymes involved in the ROS neutralization pathway include glutathione-S-transferase (GST), manganese superoxide dismutase (MnSOD) and catalase (CAT) (Hayes and Pulford, 1995). Enzymes such as MPO and endothelial nitric oxide synthase (eNOS) are involved in the generation pathway of ROS (Rehman et al., 2020). MPO catalyzes a reaction between H_2_O_2_ and chloride to generate hypochlorous acid, a potent oxidizing agent (Peng et al., 2022). A Re et al. shows that a combinatorial complex between estrogen receptor (ER)-β and endothelial nitric oxide synthase (eNOS) could repress transcription of prognostic genes that are down-regulated in prostate tumors, such as the glutathione transferase gene GSTP1 (Re et al., 2011). Kecheng Lei et al. shows that inactivation of both NQO1 and GSTP1 result in imbalanced redox homeostasis, leading to apoptosis and mitigate cancer proliferation in glioblastoma (Lei et al., 2020b). Claudia Bănescu et al. illuminats that CAT, GPX, MnSOD, and glutathione S-transferase M1 (GSTM1) and glutathione S-transferase T1 (GSTT1) gene polymorphisms are not associated with the risk of chronic myeloid leukemia (CML) except GSTP1 depending on its strong restoring ability (Bănescu et al., 2014). Therefore, in this review we focus on GSTP1, which could be a potential effective regulator in radiotherapy of cancer in GST family. Glutathione S-transferases (GST), a group of isoenzymes, were discovered in rat liver in 1960 and have gained attention for their detoxification function in catalyzing the reaction of GSH with electrophile substances (Booth et al., 1961). GSTs are found in cells mainly in the cytoplasm, mitochondria and microsomes, mainly divide into α (GSTA), π (GSTP), μ (GSTM), σ (GSTS), θ (GSTT), ζ (GSTZ), and ω (GSTO) seven isoforms. Among them, GSTP1 is the most widely studied member of the GST family (Chatterjee and Gupta, 2018; Kogawa et al., 2021). The gene encoding GSTP1 is localized on chromosome 11q13 and is approximately 3.2 kb long, which contains 9 exons and 6 introns. It has high G + C and CpG content near its 5′ end, typical of HTF (HpaII microfragment islands) (Cowell et al., 1988). GSTP1 is a phase II metabolizing enzyme that is widely found in mammalian liver, lung, kidney and other tissues. Its main function is to catalyze the binding of glutathione to various electrophilic hydrophobic substances to form water-soluble compounds for excretion from the body (Awasthi et al., 2017). Structurally, it is a dimeric protein containing 210 amino acids per subunit and two binding sites. G site specifically binds GSH and H site catalyzes the reaction of GSH with electrophile substances (FeiFei et al., 2019). GSTP1 is involved in the metabolism of various chemotherapeutic drugs and protects normal cells from carcinogens and electrophile compounds. With the continuous research on GSTP1, it has been found that besides its catalytic detoxification function, it also has various functions such as anti-apoptosis, regulation of inflammatory response, regulation of cell signaling pathways, and it is closely related to the development of tumors (van de Wetering et al., 2021). GSTP1 exists widely in the body, and its catalytic detoxification activity is believed to protect the body from carcinogenic factors. Many studies have confirmed that the expression level of GSTP1 is associated with an increased risk of various cancers. Ritchie et al. treated GSTP1 knockout mice and wild-type mice with benzopyrene, 3-methylcholanthrene, and urethane, respectively, and found that GSTP1 gene deletion increased the incidence of lung adenocarcinoma in mice exposed to these three compounds, respectively 8.3 times, 4.3 times and 8.7 times (Ritchie et al., 2007). GSTP1 may exert its protective effect on the organism by protecting normal organ tissues from carcinogenic factors due to its functions such as detoxification and regulation of inflammation. However, a large number of studies have found that the expression level of GSTP1 in most tumor cells is significantly higher than that in normal tissues, and high expression of GSTP1 is associated with poorer prognosis of tumors. Ali-Osman et al. analyzed the expression level and subcellular localization of GSTP1 in 61 primary gliomas, and analyzed the correlation between the results and tumor stage, patient age and patient survival rate. The relative risk of death in tumor patients was 3.2 times that of patients with low GSTP1 expression, and the relative risk of death in patients with GSTP1 expression in glioma nuclei was 3.9 times that in patients without GSTP1 expression in the nucleus (Ali-Osman et al., 1997). This shows that overexpression of GSTP1 protein in tumor cells and its nuclear localization are closely associated with more advanced tumor staging and worse prognosis. Pljesa-Ercegovac, M. et al. collected tumor and adjacent tissues from 84 patients with bladder transitional cell carcinoma. Through immunohistochemical analysis, they found that the apoptosis inhibitory protein Bcl-2 was highly expressed in most tumors with high GSTP1 expression, while the expression of GSTP1 was high. The level was significantly negatively correlated with the activator of apoptosis-enforcing protein caspase-3, indicating that the high expression of GSTP1 inhibited the apoptosis signaling pathway, thereby inhibiting tumor apoptosis (Pljesa-Ercegovac et al., 2011). The role of GSTP1 was explained by Savic et al.’s study on the antioxidant capacity of bladder transitional cell carcinoma. The researchers detected the activity of antioxidant enzymes in tumors and adjacent tissues of 30 patients with bladder transitional cell carcinoma, and found that γ-glutamyl cysteine synthase (γ-GCS) and glutathione in tumor tissue. The activity of peptide reductase (GR) was 4-fold and 2-fold higher than that of the paracancerous tissue, respectively, and the expression level of GSTP1 was significantly positively correlated with the activity of γ-GCS and GR. GSTP1 may participate in the regulation of cellular redox state by catalyzing the reaction of glutathione with intracellular reactive oxygen species and other electrophiles, thereby improving the antioxidant capacity of tumor cells and helping tumor cells to resist external killing factors (Savic-Radojevic et al., 2007). Our lab colleagues previously did a study on the response of GSTP1 to radiation. We found that both GSTP1 expression and its glutathione catalase activity were decreased after radiation (Lei et al., 2021b). Previous scholars have found that GSTP1 could be directly activated by NRF2 (Ikeda et al., 2002; Fang et al., 2020). At the same time, under some stress conditions (such as ionizing radiation and oxidative stress), the stress-responsive transcription factor NRF2 can induce the regulation of the SLC7A11 subunit with transport activity on System-Xc, increasing the uptake of cystine to promote further Synthesis and utilization of prototypical GSH to protect cells from ferroptosis under stressful conditions, the specific underlying mechanisms will be further explained in the outlook (Dong et al., 2021; Feng et al., 2021; Liu et al., 2022).

Till now, a specific radiosensitizer that sensitizes tumors without affecting normal tissues has not been found all over the world. Ferroptosis is a recently discovered form of cell death driven by iron-dependent lipid peroxidation which is mechanistically different from other forms of cell death. Previous studies have found that the expression of GSTP1 in tumor tissues is higher than that in normal tissues, which provides a good research entry point for us to study the potential role of GSTP1 in tumor radiotherapy through ferroptosis.

## 4 Perspective

Cells exposed to ionizing radiation may generate a large amount of reactive oxygen species and free radicals, which can lead to protein, lipid membrane and DNA damage, resulting in apoptosis, necrosis, teratogenicity or carcinogenesis (Smith et al., 2017). As a protein isoform in the glutathione S-transferase family, GSTP1 plays an important role in maintaining cellular oxidative balance, regulating cell proliferation and apoptosis. In tumor-related studies, it has been found that the high expression of GSTP1 promotes the chemoresistance of various tumors. In addition, the expression level of GSTP1 in most tumor cells is significantly higher than that in normal tissues, and high expression of GSTP1 is associated with poor prognosis of tumors (Simic et al., 2009; Fujikawa et al., 2018). Glutathione peroxidase 4 (GPX4), a potent antioxidant, utilizes glutathione as a cofactor to scavenge ROS and reduce oxidized lipid species to inhibit ferroptosis. It has been reported that glutathione metabolism in brain metastases from NSCLC is regulated by glutathione peroxidase and glutathione S-transferase; among them, GPX4 and GSTM1 are overexpressed in BM subsets, and cause massive consumption of GSH in brain metastases of lung cancer (Liu et al., 2021). Further studies find that GPX4 regulates the expression level of GSTM1 by enhancing protein stability, and the overexpression of GPX4 and its regulatory target protein GSTM1 acquires chemoresistance by inhibiting ferroptosis (Liu et al., 2021). Inhibition of GPX4 expression and its activity *in vitro* and *in vivo* enhances the anticancer effect of platinum drugs in brain metastatic cells (Liu et al., 2021). In human lung tissue, GSTP1 is the most abundant protein isoform in the GST protein family. Therefore, we speculate that GSTP1, which is a GSTM1 isoenzyme, may also be closely associated with the regulation of ferroptosis. Related studies have been listed in Table 1.

**TABLE 1:** The potential role of GSTP1 in ferroptosis pathway for tumor treatment.

Study	Year	Sample	Summary	Potential target	Possibly associated with radiotherapy
Biomimetic photosensitizer nanocrystals trigger enhanced ferroptosis for improving cancer treatment (Wu et al., 2022)	2022	Mice and HSC-3 cells	AE could induce ferroptosis by inhibiting the activity of GSTP1	LPO/GSTP1	Possible
Glutathione peroxidase 4-dependent glutathione high-consumption drives acquired platinum chemoresistance in lung cancer-derived brain (Liu et al., 2021)	2021	Immunodeficient mice and PC9‐BrM3 cells	GPX4 regulated the level of GSTM1 by protein stabilization, which is an isoenzyme with GSTP1	GSTM1	Mostly possible
Activation of mouse Pi-class glutathione S-transferase gene by Nrf2(NF-E2-related factor 2) and androgen (Ikeda et al., 2002)	2002	Mice bearing HSC-3 tumors and HepG2 cells	Nrf2 and the androgen receptor directly bind to and activate the mouse GSTP1 gene	Nrf2	Mostly possible
A targetable CoQ-FSP1 axis drives ferroptosis- and radiation-resistance in KEAP1 inactive lung cancers (Koppula et al., 2022)	2022	H1299, H23, H460, H2126 and A549	The CoQ-FSP1 axis as a key downstream effector of the KEAP1-NRF2 pathway to mediate ferroptosis -and radiation-resistance in KEAP1 deficient lung cancers	Keap1-Nrf2/FSP1-CoQ/GSTP1	Mostly possible
Activation of anti-oxidant Keap1/Nrf2 pathway modulates efficacy of dihydroartemisinin-based monotherapy and combinatory therapy with ionizing radiation (Bader et al., 2021)	2021	HCT116 cells l and NCI–H460 cells	In Keap1-wildtype cells, radiotherapy and DHA more efficiently eradicated clonogenic cells than either therapy alone	Keap1-Nrf2/GSTP1	Mostly possible
Enhanced GSTP1 expression in transitional cell carcinoma of urinary bladder is associated with altered apoptotic pathways (Pljesa-Ercegovac et al., 2011)	2011	Patients with transitional cell carcinoma	The GSTP1 expression in transitional cell carcinoma of urinary bladder is associated with altered apoptotic pathways	GSTP1	Slightly possible
Role of KEAP1/NRF2 and TP53 Mutations in Lung Squamous Cell Carcinoma Development and Radiation Resistance (Jeong et al., 2017)	2017	mice	KEAP1/NRF2 mutation status predicted risk of local recurrence after RT in non-small lung cancer patients	KEAP1/NRF2/GSTP1	Mostly possible
STK11/LKB1 Mutations in NSCLC Are Associated with KEAP1/NRF2-Dependent Radiotherapy Resistance Targetable by Glutaminase Inhibition (Sitthideatphaiboon et al., 2021)	2021	Stage III patients with NSCLC	Targeting the KEAP1/NRF2 pathway or GLS inhibition are potential approaches to radiosensitize LKB1-deficient tumors	KEAP1/NRF2/GSTP1	Mostly possible
Glutathione S-transferase-P1 expression correlates with increased antioxidant capacity in transitional cell carcinoma of the urinary bladder (Savic-Radojevic et al., 2007)	2007	Patients with transitional cell carcinoma	GSTP1 expression in tumor tissues correlated positively not only with GSH levels γ-GCS and GR activity, but also with GPX and SOD activity in TCC.	GPX/GSTP1	Mostly possible
Expression of glutathione S-transferase P1-1 in leukemic cells is regulated by inducible AP-1 binding (Duvoix et al., 2004)	2004	K562 cells	High GSTP1 gene expression could be exploited to leukaemia through binding activity to AP-1 in leukemia cells	GSTP1/AP-1	Possible
Glutathione transferases P1/P2 regulate the timing of signaling pathway activations and cell cycle progression during mouse liver regeneration (Pajaud et al., 2015)	2015	Gstp1/2 knockout mice in C57BL6/J	The invalidation of Gstp1/p2 affects multiple key events of the hepatocyte cell cycle	GSTP1	Slightly possible
Regulation of glutathione S-transferase P1-1 gene expression by NF-kappaB in tumor necrosis factor alpha-treated K562 leukemia cells (Morceau et al., 2004)	2004	K562 cell	The regulation of the GSTP1-1 gene expression in the K562 cell line by NF-kappaB and TNFα	GSTP1	Slightly possible
GSTP1 Loss results in accumulation of oxidative DNA base damage and promotes prostate cancer cell survival following exposure to protracted oxidative stress (Mian et al., 2016)	2016	LNCaP cells	Silencing of GSTP1 in prostate cancer results in enhanced survival and accumulation of potentially promutagenic DNA adducts following exposure of cells to protracted oxidative injury	GSTP1	Mostly possible

AE, aloe-emodin; LPO, lipid peroxidation; FSP1, ferroptosis suppressor protein 1; CoQ, coenzyme Q(10); GSTM1, Glutathione S-transferase M1; Keap1, kelch-like ECH associated protein 1; Nrf2, nuclear factor erythroid 2-related factor 2; RT, radiation therapy; GSTP1, Glutathione S-transferase P1; GSH, glutathione; GPX4, glutathione peroxidase 4; LKB1, live kinase B1; γ-GCS, γ-glutamyl cysteine synthase; SOD, superoxide dismutase; TCC, transitional cell carcinoma; TNFα, tumor necrosis factor alpha.

Ferroptosis is an iron-dependent lipid peroxidation-mediated cell death. Researchers find that autophagy inhibitors can protect HepG2 cells from alcohol-induced ferroptosis by activating the p62-Keap1-Nrf2 pathway (Zhao et al., 2021). It has also been found that Keap1/Nrf2 mutation status predicts the risk of local recurrence after radiotherapy in NSCLC patients, and Keap1/Nrf2 mutant lung cancers may be radiotherapy resistant to radaition due to enhanced expression of ROS clearance and detoxification pathways (Jeong et al., 2017). Keap1 is a negative regulator of Nrf2, and Nrf2 is a major effector of the ARE system. Activation of the ARE system through negative regulation of Keap1 protein induces the expression of a range of antioxidant genes, including Nrf2 and GSTP 1 (Fang et al., 2020; Umamaheswari et al., 2021). The function of GSTP1 is to catalyze the binding of GSH to various electrophilic hydrophobic substances to form water-soluble compounds for excretion from the body (Ikeda et al., 2002; Cui et al., 2020). Lei et al. further demonstrats that Keap1 deficiency in lung cancer cells promotes radioresistance in lung squamous cell carcinoma in part through SLC7A11 inhibition of ferroptosis (Lei et al., 2020a). Interestingly, it is found that GSTP1 expression is regulated by the Keap1-Nrf2-ARE pathway and GSTP1 catalyzes the S-glutathionylation of cysteine residues of Keap1 protein, while S-glutathionylation of Keap1 leads to Nrf2 activation and increases the expression of GSTP1 (Carvalho et al., 2016). It has also been found that the promoter of the mouse GSTP1 gene contains at least three Nrf2 binding sites, demonstrating that Nrf2 directly activates the gene and that GSTP1 gene expression directly affects the Nrf2-dependent response to the hormone diselenide (Ikeda et al., 2002; Bartolini et al., 2015).

Therefore, we speculate that lung cancer cells might form a GSTP1-Keap1-Nrf2 positive feedback loop under ionizing radiation or oxidative stress, and play an anti-oxidative damage effect. At the same time, SLC7A11 is up-regulated by the transcription of Nrf2, thereby increasing the resistance to ionizing radiation. GSTP1 catalyzes the reaction of glutathione with electrophiles, including intracellular reactive oxygen species, hydroxyl radicals, and inhibits its oxidation of polyunsaturated fatty acids on the cell membrane to fight ferroptosis. In addition, GSTP1 may also interact with GPX4 to play a synergistic role in inhibiting the occurrence of ferroptosis, thereby enhancing the radioresistance of tumors. The potential mechanism is shown as following (Figure 1). Moreover, GSTP1 is involved in ferroptosis regulatory mechanisms possibly similar to GPX4 as part of the ferroptosis pathway. Targeting downregulation of GSTP1 expression under tumor radiotherapy would increase radiosensitivity of lung tumors and thus promoting radiation-induced ferroptosis. On the one hand, it may act from promoting lipid metabolism through the ferroptosis execution system, on the other hand, it may weaken the ferroptosis defense system by reduce the ability of cells to use GSH to counteract ROS. In addition, radiation may make the interaction between GSTP1 and GPX4 decreased, which further promotes the occurrence of ferroptosis. However, the exact mechanism still need to be confirmed by further experiments.

**FIGURE 1:** The potential role of GSTP1 and its mechanisms of ferroptosis in radiotherapy. Keap1-Nrf2-GSTP1 positive feedback loop interacts with GPX4 and SLC7A11 which are the core proteins in ferroptosis pathway under radiation. Their interactions affect lipid peroxidation, thus inhibiting the occurrence of ferroptosis (Liu et al., 2021; Wu et al., 2022). (IR: ionizing radiation; Keap1: kelch-like ECH associated protein 1; Nrf2: nuclear factor erythroid 2-related factor 2; GSTP1: Glutathione S-transferase P1; GSH: glutathione; GPX4: glutathione peroxidase 4).

Although no experimental studies have shown that GSTP1 plays a key role in the radiosensitization of ferroptosis in lung cancer, previous studies by our group showed that the levels of MDA, the lipid peroxide breakdown product, were significantly increased in cells with knockdown of GSTP1 after radiation treatment. In addition, multiple studies have shown that higher serum iron concentrations and ferritin levels are positively associated with lung cancer morbidity and mortality. It also laid a theoretical foundation for our subsequent exploration of the mechanism by which GSTP1 may protect lung cancer cells and inhibit ferroptosis after tumor radiation therapy.

## 5 Conclusion

In conclusion, GSTP1 may be a novel negative regulator of ferroptosis other than GPX4, may play an important role in lung cancer radiotherapy by inhibiting ferroptosis. The reasons are as follows. Firstly, as a potent antioxidant, GPX4 utilizes glutathione as a cofactor to scavenge ROS and reduces oxidized lipid species to inhibit ferroptosis (Friedmann Angeli et al., 2014; Stockwell et al., 2020). It has been reported that glutathione metabolism in brain metastases from NSCLC is regulated by glutathione peroxidase and glutathione S-transferase; among them, GPX4 and GSTM1 are overexpressed in BM subsets, and cause massive consumption of GSH in brain metastases of lung cancer (Liu et al., 2021). Further studies find that GPX4 regulates the expression level of GSTM1 by enhancing protein stability, and the overexpression of GPX4 and its regulatory target protein GSTM1 acquires chemoresistance by inhibiting ferroptosis. Inhibition of GPX4 expression and its activity *in vitro* and *in vivo* enhances the anticancer effect of platinum drugs in brain metastatic cells (Liu et al., 2021). Secondly, as a member of GSTs, GSTP1 could participate in the metabolism of lipids and DNA products derived from oxidative stress. The core of ferroptosis is the excessive accumulation of intracellular lipid peroxides, which is caused by the imbalance of lipid metabolism from various causes (Luo et al., 2022). Besides, Zhao et al. find that GSTP1 is a key protein for ferroptosis. And the photosensitizer aloe-emodin (AE) could induce cellular ferroptosis based on its specific inhibiting activity to GSTP1 (Wu et al., 2022). The underlying mechanism of GSTP1 in the induction of ferroptosis in lung cancer radiotherapy has been proposed in a hypothetical pathway map (Figure 1). In addition, although relevant studies have shown that GSTP1 is closely related to the occurrence and development of tumors, there is no specific experimental study to prove the role and mechanism of GSTP1 in ferroptosis radiotherapy. This provides us with a research entry point to develop better personalized treatment strategies for the clinic. So far, there are multiple evidences that targeting GSTP1 can have a synergistic effect with chemotherapeutic drugs, but there is no correlation between GSTP1 and radiation-induced ferroptosis. If the changes of GSTP1 protein expression or activity can be controlled, thereby increasing the ferroptosis effect of radiotherapy on lung tissue tumors, while reducing radiation damage to normal lung tissue, it has extremely important medical significance for the treatment and prognosis of thoracic tumor patients. This is the core purpose of this review.
